The article "Alga Ecklonia bicyclis, Tribulus terrestris, and Glucosamine Oligosaccharide Improve Erectile Function, Sexual Quality of Life, and Ejaculation Function in Patients with Moderate Mild-Moderate Erectile Dysfunction: A Prospective, Randomized, Placebo-Controlled, Single-Blinded Study" was published in 2014. Journal: Biomed Res Int.

# Alga *Ecklonia bicyclis*, *Tribulus terrestris*, and Glucosamine Oligosaccharide Improve Erectile Function, Sexual Quality of Life, and Ejaculation Function in Patients with Moderate Mild-Moderate Erectile Dysfunction: A Prospective, Randomized, Placebo-Controlled, Single-Blinded Study

**DOI:** 10.1155/2014/121396

**Published:** 2014-07-20

**Authors:** Salvatore Sansalone, Rosario Leonardi, Gabriele Antonini, Antonio Vitarelli, Giuseppe Vespasiani, Dragoslav Basic, Giuseppe Morgia, Sebastiano Cimino, Giorgio Ivan Russo

**Affiliations:** ^1^Department of Experimental Medicine and Surgery, Tor Vergata University of Rome, Rome, Italy; ^2^Centro Uro Andrologico, Acireale, Italy; ^3^Department of Urology “U. Bracci”, La Sapienza University of Rome, Rome, Italy; ^4^Urologia Universitaria II, Azienda Ospedaliera Policlinico Bari, Bari, Italy; ^5^Clinic of Urology, Clinical Center Nis, Nis, Serbia; ^6^School of Medicine Policlinico Hospital, Department of Urology, University of Catania, Catania, Italy

## Abstract

We aimed to evaluate the efficacy of oral therapy with alga *Ecklonia bicyclis*, *Tribulus terrestris*, and glucosamine oligosaccharide (Tradamix TX1000) in patients with erectile dysfunction (ED) at 3 months of follow-up. From January 2013 to September 2013, 177 patients diagnosed with mild-moderate ED (IIEF-EF < 26) were enrolled in this multicenter, single-blinded, placebo-controlled study and randomized in Group A (Tradamix, *n* = 87) and Group B (placebo, *n* = 90). Penile color Doppler ultrasound measures, IIEF-15 questionnaire, male sexual health questionnaire-ejaculation disorder (MSHQ-EjD), and sexual quality of life (SQoL-M) were collected. We observed significant changes of the IIEF-15 in Group A (mean difference: 11.54; *P* < 0.05) at 3 months versus Group B (*P* < 0.05). PSV (*P* < 0.05), IIEF-intercourse satisfaction (*P* < 0.05), IIEF-orgasmic function (mean *P* < 0.05), IIEF-sexual desire (*P* < 0.05), IIEF-overall satisfaction (*P* < 0.05), MSHQ-EjD (mean difference: 1.21; *P* < 0.05), and SQoL-M (mean difference: 10.2; *P* < 0.05) were significantly changed in Group A versus baseline and Group B. Patients with moderate arterial dysfunction showed significant increase of PSV (*P* < 0.05), IIEF-EF (*P* < 0.05), MSHQ-EjD (*P* < 0.05), and SQoL-M (*P* < 0.05) in Group A. Therapy with Tradamix improves erectile and ejaculation function and sexual quality of life in patients with mild-moderate ED and in particular for those with moderate arterial dysfunction.

## 1. Introduction

All over the world, erectile dysfunction (ED) is considered one of the most diffuse sexual disorders. The prevalence rate of ED increases with age and with concomitant morbidities. To this regard, erectile dysfunction (ED) has progressively emerged as an important indicator of men's overall health, due to the very closed relationship to concomitant comorbidities [1–4].

The article "Alga Ecklonia bicyclis, Tribulus terrestris, and Glucosamine Oligosaccharide Improve Erectile Function, Sexual Quality of Life, and Ejaculation Function in Patients with Moderate Mild-Moderate Erectile Dysfunction: A Prospective, Randomized, Placebo-Controlled, Single-Blinded Study" was published in 2014. Journal: Biomed Res Int.

Several observational studies recently demonstrated that ED is associated with different comorbid condition and overall poorer male health [5, 6], but also ED may significantly increase the risk of cardiovascular disease (CVD), coronary heart disease, stroke [7], and all-cause mortality [8–11], and this increase is probably independent from conventional cardiovascular risk factors [9] and glycometabolic control [12].

Based on these considerations, phosphodiesterase-5 inhibitors (PDE5-i) have become the most popular treatment and are currently the first line monotherapy for ED [13].

However, it should be taken into account that some patients with complex ED may not be responders to PDE5-I monotherapy [14]. Furthermore, this category of drugs is not depicted from side effects that could impair pharmacological adherence.

The most common reported side effects are headache, muscular pains, hot flushes, tearing, and so on that can affect normal sexual intercourse [15]. It is also generally known that ED may be associated with serum total testosterone (TT) alterations. In fact, TT in men begins to decline in the late third or early fourth decade and diminish at a constant rate thereafter [16].

In this general context, studies on natural compounds have been conducted with the intention to limit side effects and to maintain efficacy [17, 18]. A new natural compound made of alga* Ecklonia bicyclis*,* Tribulus terrestris*, and glucosamine oligosaccharide has been diffused in order to improve male sexual function in elderly men, particularly libido and possible erectile dysfunction.* Ecklonia bicyclis* has radical scavenger activity 10–100 times more powerful than any other polifenol terrestris plants, which have only 3-4 phenolic and rings that are commonly considered among the most effective antioxidant molecules. The protodioscin is a steroidal saponin, which is about 90% of the extract obtained from aerial parts of* Tribulus terrestris*. Thanks to its particular steroidal structure it has an androgen mimetic action, binding and activating the receptor of testosterone. So this substance is able to increase the endogenous production of testosterone, dihydrotestosterone, hormone luteinizing hormone (LH), dehydroepiandrosterone (DHEA), and dehydroepiandrosterone sulfate (DHEAS).

glucosamine oligosaccharide acts both on nonadrenergic and noncholinergic system (NANC) and on endothelial cell system as a strong nitric oxide synthetase (NOS) simulator [16].

The article "Alga Ecklonia bicyclis, Tribulus terrestris, and Glucosamine Oligosaccharide Improve Erectile Function, Sexual Quality of Life, and Ejaculation Function in Patients with Moderate Mild-Moderate Erectile Dysfunction: A Prospective, Randomized, Placebo-Controlled, Single-Blinded Study" was published in 2014. Journal: Biomed Res Int.

The aim of this prospective multicenter randomized, single-blinded, placebo-controlled study was to evaluate the efficacy and tolerability of the combination therapy with alga* Ecklonia bicyclis*,* Tribulus terrestris*, and glucosamine oligosaccharide in patients mild-moderate erectile dysfunction at 3 months of follow-up.

## 2. Patients and Methods

From January 2013 to September 2013, 214 patients diagnosed with mild-moderate ED (IIEF-EF < 26) were entered in this prospective multicenter randomized, single-blinded, placebo-controlled study. All subjects gave written informed consent before entering the study, which was conducted in accordance with the Declaration of Helsinki, and the Human Ethics Committee approved the study protocol (Serbian Ministry Of Education and Science, Grant No175092). All patients underwent preliminary assessment including a detailed medical and sexual history to evaluate the presence of risk factors such as diabetes mellitus, hypertension, dyslipidaemia, and smoking. All subjects were self-administered the IIEF-15 item questionnaire and the Male Sexual Health Questionnaire-Ejaculation Disorder (MSHQ-EjD) and sexual quality of life instrument for men (SQoL-M).

The primary inclusion criteria were a minimum age of 18 years, a diagnosis of nonendocrinological ED according to the National Institutes of Health statement on ED, 1 naïve to treatment for ED, a stable heterosexual relationship for at least the previous 6 months, and a steady relationship with the same female partner.

Exclusion criteria were as follows: severe ED (IIEF-EF < 11), previous medical or surgical treatments for ED, any medical treatment for sexual dysfunction before or during the study, congenital or acquired penile curvature or chordee with hypospadias, age >75 years, hypogonadism (total testosterone level of <8 nmol or serum testosterone in the range of 8–11 nM and free testosterone <220 pmol, assessed at least on two occasions), and end diastolic velocity (EDV) >5 cm/s at penile color doppler ultrasound (CDU).

All patients were also subjected to a thorough physical examination. To be able to exclude organic sexual dysfunctions and other underlying illnesses, fasting blood glucose level, urinalysis, complete blood count, sex hormones, and prolactin levels were measured.

All measurements were conducted by a single physician unaware of the treatment status.

Patients were randomized according to a computer generated random sequence with a 1 : 1 ratio in two treatment groups, namely, Group A and Group B. The first group received one tablet orally twice a day for 3 months and one tablet consisted of 300 mg of alga* Ecklonia bicyclis*, 450 mg of* Tribulus terrestris* and 250 mg of glucosamine oligosaccharide (Tradamix TX1000, Tradapharma Sagl, Switzerland), while the second received one table twice a day for 3 months of placebo. We monitored adverse events on the light of common terminology criteria for adverse events (CTCAE) guidelines.

The article "Alga Ecklonia bicyclis, Tribulus terrestris, and Glucosamine Oligosaccharide Improve Erectile Function, Sexual Quality of Life, and Ejaculation Function in Patients with Moderate Mild-Moderate Erectile Dysfunction: A Prospective, Randomized, Placebo-Controlled, Single-Blinded Study" was published in 2014. Journal: Biomed Res Int.

### 2.1. Main Outcome Measures

The primary efficacy outcome was the change from baseline to end point (3 months) for the IIEF-15. Secondary outcomes were the change from baseline to end point of IIEF-15 subscore, MSHQ-EJD, SQoL-M, and PSV. Safety assessments included treatment-emergent adverse events (TEAEs), serious AEs (SAEs), and orthostatic vital signs (blood pressure and heart rate).

### 2.2. Study Population

The study sample of 170 was powered for an approximately 10-point difference of the IIEF-15 using a two-sided type I error = 0.05 and type II error = 0.1 (90% power), requiring patients per group. The maximum sample size was set to 100 subjects per group, allowing for a 15% dropout rate.

### 2.3. Statistical Analysis

At baseline, the independent sample 2-tailed* t*-test was used to compare variables. For categorical parameters, chi-square test was applied. Changes from baseline to end of therapy were analysed using ranked one-way analysis of variance (ANOVA) with a term for treatment group. According to the penile Doppler ultrasound analysis, patients were divided into three categories: normal arterial function (NAF) (PSV ≥ 35 cm/s), moderate arterial dysfunction (MAD) (PSV ≥ 25 and <35 cm/s), and severe arterial dysfunction (SAD) (PSV < 25 cm/s). Treatment group differences for primary and secondary end points were determined using post hoc analysis. Data were reported as means ± standard deviation (SD) or median and nominal *P* values were presented. For all statistical comparisons, significance was considered as *P* < 0.05.

## 3. Results

Table 1 lists the baseline characteristics of patients enrolled. Of the 214 patients, 14 (6.54%) were excluded from the study because they did not meet the entry criteria. Of the 200 patients randomized, 87 and 90 subjects in Group A and in Group B completed the study protocol. The flow chart of this study is presented in Figure 1.

### 3.1. Main Outcome Measures

Table 2 lists the mean change differences from baseline to 3 months relative to main outcome measures. When concerning the primary endpoint of this study, we observed significant changes of the IIEF-15 in Group A (mean difference: 11.54; *P* < 0.05) at 3 months versus Group B at the intergroup analysis (mean difference: 10.22; *P* < 0.05). In Group A, significant differences from baseline to last follow-up were observed relative to PSV (mean difference: 1.36 cm/s; *P* < 0.05), IIEF-IS (mean difference: 1.72; *P* < 0.05), IIEF-OF (mean difference: 2.2; *P* < 0.05), IIEF-SD (mean difference: 1.03; *P* < 0.05), IIEF-OS (mean difference: 2.51; *P* < 0.05), MSHQ-EjD (mean difference: 1.21; *P* < 0.05), and SQoL-M (mean difference: 10.2; *P* < 0.05). In Group A, patients with moderate arterial dysfunction showed significant increase of IIEF-EF (mean difference: 1.82; *P* < 0.05), PSV (mean difference: 1.56; *P* < 0.05), MSHQ-EjD (mean difference: 1.23; *P* < 0.05), and SQoL-M (mean difference: 11.65; *P* < 0.05) from baseline to 3 months. Significant differences were found at the intergroup analysis when considering previous outcome measures (Table 2) and (Figure 2). Patients with normal arterial function and with severe arterial dysfunction of Group A did not report improvement of penile CDU measures after treatment. When considering serum TT and EDV, both groups did not show any difference after 3 months. All subjects included in the study protocol tolerated treatments, and none reported adverse events.

The article "Alga Ecklonia bicyclis, Tribulus terrestris, and Glucosamine Oligosaccharide Improve Erectile Function, Sexual Quality of Life, and Ejaculation Function in Patients with Moderate Mild-Moderate Erectile Dysfunction: A Prospective, Randomized, Placebo-Controlled, Single-Blinded Study" was published in 2014. Journal: Biomed Res Int.

## 4. Discussion

Several studies have established that reactive oxygen ROS, especially superoxide anion and hydrogen peroxide, are important signaling molecules in cardiovascular cells [19, 20]. Enhanced superoxide production increases NO inactivation and leads to an accumulation of peroxynitrites and hydrogen peroxide [21]. ROS participate in growth, apoptosis, and the migration of vascular smooth muscle cells, in the modulation of endothelial function (including endothelium-dependent relaxation and expression of a proinflammatory phenotype), and in the modification of the extracellular matrix [22–24]. All of these events play important roles in endothelial dysfunction, suggesting that the sources of ROS and the signaling pathways that they modify may represent important therapeutic targets [25].

All these findings have determined the diffusion of several herbal extract with the intention of targeting previous pathways.

An interesting in vivo and in vitro animal investigations of a mixture of herbal extracts from* T. terrestris* and* C. officinalis* were conducted to investigate their relaxation effects and the mechanisms of action on penile erection.* T. terrestris* extract,* C. officinalis* extract, and the mixture of both extracts showed concentration-dependent relaxation effects of the corpus cavernosum. Therefore, endothelium appears to be an important location of action of* T. terrestris* extract, functioning in relaxation mainly via NOS and exhibited relaxation effects mainly through cAMP and partly through cGMP [26].

It can be supposed that because herbal extracts do not contain a single ingredient but are a combination of multiple compounds, it would not be appropriate to expect a mechanism of action similar to that of a single compound such as a PDE-5 inhibitor.* C. officinalis* extract appears to exhibit relaxation effects by acting directly on the smooth muscle cells of the CC, not through the above pathway. With the administration of the mixture of extracts, cAMP concentration in the CC increased significantly. Based on the previous results, the extracts studied appear to exhibit relaxation effects on the CC mainly through cAMP and partly through cGMP.

The article "Alga Ecklonia bicyclis, Tribulus terrestris, and Glucosamine Oligosaccharide Improve Erectile Function, Sexual Quality of Life, and Ejaculation Function in Patients with Moderate Mild-Moderate Erectile Dysfunction: A Prospective, Randomized, Placebo-Controlled, Single-Blinded Study" was published in 2014. Journal: Biomed Res Int.

This can be explained by the multiple mechanism of action of these compounds on several targets with the consequent therapeutical efficacy.

Based on our results and considering all subdomains of 15-question International Index of Erectile Function, therapy with multiple antioxidants was significantly superior in improving intercourse satisfaction, sexual desire, orgasmic function, and overall satisfaction. In fact, it should be noted that the severity of penile curvature or deformity may significantly contribute to man's inability to have intercourse.

Furthermore, patients referred the improvement of ejaculation and quality of life, as assessed by the MSHQ-EjD and the SQoL-M), although there was a short follow-up.

This new natural compound is thought to play an important double role (therapeutic and antiaging), on cavernous tissue, by acting on the etiopathogenetic aspects of ED, mainly the microstructural alteration of the corpus cavernosum tissues, following inflammation and/or oxidative damage [16].

We suppose that this combination of natural compounds may strength the efficacy of the single component, the* Ecklonia bicyclis* by a radical scavenger activity, the protodioscin by binding and activating the receptor of testosterone, and the glucosamine oligosaccharide, by acting on the nonadrenergic and noncholinergic system (NANC) and on the endothelial cell system as a strong nitric oxide synthetase (NOS) stimulator, thus improving the concentration of nitric oxide (NO) in the smooth cells inside the corpus cavernosum.

These considerations may explain the significant changes of IIEF-EF, MSHQ-EjD, PSV, and SQoL-M in Group A for men with moderate arterial penile dysfunction. We can affirm in fact that those with severe arterial dysfunction may not have benefits from therapy with natural compounds, since their ED was worse.

Penile CDU evaluation in ED has a significant role in determining the cause of ED. Arteriogenic ED or arterial insufficiency is diagnosed when PSV is <25 cm/s, with angiographic correlation showing that a PSV threshold of 25 cm/s has 92% accuracy in diagnosis of arterial integrity. Penile CDU represents an accurate tool to investigate cavernous artery inflow and venous leakage frequently used for assessing the efficacy of several genitourethral reconstruction surgical techniques, in patients who underwent urethroplasty, peyronie's disease related surgery, or penile revascularization [27, 28].

The article "Alga Ecklonia bicyclis, Tribulus terrestris, and Glucosamine Oligosaccharide Improve Erectile Function, Sexual Quality of Life, and Ejaculation Function in Patients with Moderate Mild-Moderate Erectile Dysfunction: A Prospective, Randomized, Placebo-Controlled, Single-Blinded Study" was published in 2014. Journal: Biomed Res Int.

In this context, although the prevalence of ED before and after genitourethral reconstruction surgeries has not been correctly investigated, it may affect the expectancy of these techniques with failed results.

Although our population study was represented by subjects who did not underwent previous genitourethral reconstruction surgeries, we may suggest with caution to use oral therapy with alga* Ecklonia bicyclis*,* Tribulus terrestris*, and glucosamine oligosaccharide with the intention to ameliorate penile CDU in patients eligible for penile surgery.

However, this study is not depicted from limitations. First of all a longer follow-up would have added more information about the efficacy and its maintenance over the time. Second, ED was assessed by questionnaire and penile Doppler ultrasound and ejaculation function by the MSHQ-ED. Certainly, some more diagnostic procedures would have been beneficial. In conclusion, oral therapy with alga* Ecklonia bicyclis*,* Tribulus terrestris*, and glucosamine oligosaccharide has significant advantages in patients with mild-moderate ED, by improving intercourse satisfaction, sexual desire, orgasmic function, overall satisfaction, ejaculation function, and quality of life. Further clinical study, involving a general population eligible for genitourethral reconstruction surgery may offer new insight about the efficacy of combination with alga* Ecklonia bicyclis*,* Tribulus terrestris*, and glucosamine oligosaccharide.

## 5. Conclusion

Patients affected by mild-moderate ED may significantly benefit from oral therapy with alga* Ecklonia bicyclis*,* Tribulus terrestris*, and glucosamine oligosaccharide by improving sexual and ejaculation function and sexual quality of life. In particular, those with moderate arterial dysfunction, considered as a peak systolic velocity (PSV) ≥25 and <35 cm/s, may significantly benefit from this therapy thanks to the improvement of IIEF-EF, MSHQ, SQoL-M, and PSV.

## Figures and Tables

**Figure 1:** Disposition of subjects. Subject consolidated standards of reporting trials (CONSORT) diagram.

**Figure 2:** Mean changes from baseline to 3 months for International Index of Erectile Function domain (^a^ *P* < 0.05, versus baseline; ^b^ *P* < 0.05, versus Group B).

**Table 1:** Baseline characteristics of patients enrolled.

	Group A (TRADAMIX TX 1000)	Group B (Placebo)
Number of patients	87	90
Age (yr), mean ± SD	63.92 ± 9.3	65.37 ± 8.81
BMI (Kg/m²), mean ± SD	26.36 ± 3.0	25.2 ± 3.5
Hypertension, *n* (%)	40 (44.94)	42 (46.66)
Dyslipidemia, *n* (%)	24 (27.58)	2 (25.5)
Diabetes, *n* (%)	17 (19.54)	18 (20.0)
Total testosterone, mean	14.69 ± 1.25	13.26 ± 1.02
Smoking habit, *n* (%)	40 (39.21)	38 (38.0)
IIEF-EF, mean ± SD	21.16 ± 4.08	20.71 ± 3.77
IIEF-IS, mean ± SD	5.80 ± 2.07	6.06 ± 1.91
IIEF-OF, mean ± SD	5.11 ± 1.23	5.37 ± 1.37
IIEF-SD, mean ± SD	7.97 ± 1.69	7.80 ± 1.81
IIEF-OS, mean ± SD	4.89 ± 1.66	4.86 ± 1.44
MSHQ-EjD, mean ± SD	14.89 ± 3.09	14.50 ± 2.87
SQoL-M, mean ± SD	54.21 ± 2.11	55.87 ± 2.35
PSV, mean ± SD	31.52 ± 6.60	30.02 ± 5.56
EDV, mean ± SD	1.5 ± 1.0	1.2 ± 2.0
Normal arterial function (PSV ≥ 35 cm/s), *n* (%)	36 (35.3)	30 (33.3)
Moderate arterial dysfunction (PSV ≥ 25 and <35 cm/s), *n* (%)	31 (30.4)	29 (32.2)
Severe arterial dysfunction (PSV < 25 cm/s), *n* (%)	20 (19.6)	22 (24.4)

BMI = Body Mass Index; IIEF-EF = International Index of Erectile Function-Erectile Function; IIEF-IS = International Index of Erectile Function-Intercourse Satisfaction; IIEF-OF = International Index of Erectile Function-Orgasmic Function; IIEF-SD = International Index of Erectile Function-Sexual Desire; IIEF-OS = International Index of Erectile Function-Overall Satisfaction; MSHS-EJD = Male Sexual Health Questionnaire-Ejaculation Disorder; SQoL-M = sexual quality of life instrument for men; PSV = peak systolic velocity; EDV = end diastolic velocity.

The article "Alga Ecklonia bicyclis, Tribulus terrestris, and Glucosamine Oligosaccharide Improve Erectile Function, Sexual Quality of Life, and Ejaculation Function in Patients with Moderate Mild-Moderate Erectile Dysfunction: A Prospective, Randomized, Placebo-Controlled, Single-Blinded Study" was published in 2014. Journal: Biomed Res Int.

**Table 2:** Mean changes from baseline to 3 months for primary and secondary outcomes.

	Group A	Group B
IIEF-15, mean ± SD	11.54 ± 2.47^a,b^	1.32 ± 2.67
IIEF-EF, mean ± SD	0.35 ± 1.42	0.04 ± 1.00
IIEF-IS, mean ± SD	1.72 ± 1.63^a,b^	0.05 ± 2.15
IIEF-OF, mean ± SD	2.20 ± 1.51^a,b^	0.08 ± 1.77
IIEF-SD, mean ± SD	1.03 ± 1.35^a,b^	0.41 ± 0.34
IIEF-OS, mean ± SD	2.51 ± 1.45^a,b^	0.57 ± 0.39
MSHQ-EjD, mean ± SD	1.21 ± 2.03^a,b^	0.24 ± 1.07
SQoL-M, mean ± SD	10.20 ± 3.77^a,b^	1.24 ± 2.53
PSV (cm/s), mean ± SD	1.36 ± 0.75^a,b^	0.21 ± 0.44
EDV (cm/s), mean ± SD	0.24 ± 1.0	0.31 ± 0.9
Total testosterone (nmol/L), mean ± SD	14.26 ± 2.05	13.31 ± 1.32
Normal arterial function (PSV ≥35 cm/s) subgroup		
IIEF-EF, mean ± SD	0.94 ± 3.68	0.10 ± 4.10
PSV (cm/s), mean ± SD	0.16 ± 0.75	0.10 ± 0.87
MSHQ-EJD, mean ± SD	1.41 ± 1.85^a,b^	0.32 ± 1.54
SQoL-M, mean ± SD	8.76 ± 3.65	1.41 ± 3.21
Moderate arterial dysfunction (PSV ≥25 and <35 cm/s) subgroup		
IIEF-EF, mean ± SD	1.82 ± 3.08^a,b^	0.16 ± 2.69
PSV (cm/s), mean ± SD	1.56 ± 0.82^a,b^	0.23 ± 0.63
MSHQ-EJD, mean ± SD	1.23 ± 1.84^a,b^	0.11 ± 1.52
SQoL-M, mean ± SD	11.65 ± 3.12^a,b^	1.18 ± 2.87
Severe arterial dysfunction (PSV <25 cm/s) subgroup		
IIEF-EF, mean ± SD	0.54 ± 2.77	0.23 ± 2.41
PSV (cm/s), mean ± SD	0.05 ± 0.52	0.09 ± 0.74
MSHQ-EJD, mean ± SD	0.90 ± 2.56	0.25 ± 2.31
SQoL-M, mean ± SD	2.43 ± 2.89	1.21 ± 3.44

^a^ *P* < 0.05 versus baseline; ^b^ *P* < 0.05 versus Group B.
